# Cardiac Magnetic Resonance Images Superresolution via Multichannel Residual Attention Networks

**DOI:** 10.1155/2021/8214304

**Published:** 2021-08-12

**Authors:** Defu Qiu, Yuhu Cheng, Xuesong Wang

**Affiliations:** ^1^Engineering Research Center of Intelligent Control for Underground Space, Ministry of Education, China University of Mining and Technology, Xuzhou 221116, China; ^2^School of Information and Control Engineering, China University of Mining and Technology, Xuzhou 221116, China

## Abstract

The deep neural network has achieved good results in medical image superresolution. However, due to the medical equipment limitations and the complexity of the human body structure, it is difficult to reconstruct clear cardiac magnetic resonance (CMR) superresolution images. To reconstruct clearer CMR images, we propose a CMR image superresolution (SR) algorithm based on multichannel residual attention networks (MCRN), which uses the idea of residual learning to alleviate the difficulty of training and fully explore the feature information of the image and uses the back-projection learning mechanism to learn the interdependence between high-resolution images and low-resolution images. Furthermore, the MCRN model introduces an attention mechanism to dynamically allocate each feature map with different attention resources to discover more high-frequency information and learn the dependency between each channel of the feature map. Extensive benchmark evaluation shows that compared with state-of-the-art image SR methods, our MCRN algorithm not only improves the objective index significantly but also provides richer texture information for the reconstructed CMR images, and our MCRN algorithm is better than the Bicubic algorithm in evaluating the information entropy and average gradient of the reconstructed image quality.

## 1. Introduction

The heart is the core organ that ensures the continuation of human life and metabolism. Its main function is to provide power for blood flow in the body through the contraction pressure of the heart muscle. Cardiac magnetic resonance (CMR) imaging [1] is an important technique for the functional analysis of the heart. It is suitable for the accurate assessment and analysis of the local and global function of cardiac tissue structures, and it plays an important role in assisting physicians in diagnosis and treatment and improving diagnostic accuracy. The CMR imaging can perform multiphase imaging in the time domain to form a dynamic image sequence of the cardiac cycle. Based on the imaging results, cardiac function evaluation indicators, such as ejection fraction, myocardial mass, and myocardial thickness, can be obtained, which is convenient for medical experts to analyze the systolic function of the heart and diagnose diseases [2–4]. However, the CMR images are very different from conventional images. Due to the performance limitations of medical equipment and the complexity of human body structure, the CMR images often have very low resolution and have a lot of noise, which directly affects expert judgment of heart disease [5]. Therefore, there are an urgent need and practical significance for the study of image SR reconstruction algorithms for CMR images.

With the deepening of research on SR tasks, many SR algorithms have emerged. These algorithms can be roughly divided into three categories: interpolation-based methods [6], reconstruction-based methods [7], and learning-based methods [8]. Since deep learning has achieved outstanding performance in various fields of computer vision in recent years, learning-based SR methods have also become a hot spot in superresolution technology research, whose purpose to recover high-resolution (HR) images from low-resolution (LR) images. Dong et al. [9] proposed the SR convolutional neural network (SRCNN) and achieved excellent performance. On this basis, Dong et al. [10] improved the SRCNN algorithm and proposed the fast SR convolutional neural networks (FSRCNN) to accelerate the training speed of the network. Kim et al. [11] proposed the superresolution using very deep convolutional network (VDSR), which uses the idea of residual error to alleviate the problem of gradient disappearance or gradient explosion. Since only the high frequency of the image is learned information, the convergence speed is significantly improved; at the same time, a larger receptive field is used in VDSR to improve the effect and multiscale issues considered in the single model.

After that, Kim et al. [12] considered the problem of parameter scale and proposed the deep recursive convolutional network (DRCN), which uses a recursive network structure to share parameters between network structures, which effectively reduces the difficulty of training; in addition, the authors also use skip connection and integration strategies to further improve performance. Subsequently, Shi et al. [13] proposed the efficient subpixel convolutional neural network (ESPCN), which uses LR images as input and uses subpixel convolutional layers at the back end of the network structure to implicitly map LR images to HR images, effectively reducing computational complexity and improving reconstruction efficiency. Lai et al. [14] proposed the Laplacian pyramid networks (LapSRN), the idea of Laplace pyramid is introduced into deep learning, and the experimental results prove the superiority of step-by-step sampling operation. In addition, the residual results predicted at each level are monitored during the training process, which further improves the performance. Lim et al. [15] proposed the enhanced deep residual networks for single image superresolution (EDSR) by removing the redundant modules in the literature [16] and using the L1 norm as the loss function. Zhang et al. [17] proposed the residual channel attention network (RCAN), by using the channel attention mechanism, a feature channel with rich information can be selected. The above network structures are mostly feed-forward structures, ignoring the interdependence of HR images and LR images and the error when upsampling LR images. In addition, Haris et al. [18] proposed the deep back-projection networks (DBPN), which uses the upsampling interconnection strategy and error feedback mechanism to learn the mutual mapping relationship between HR and LR and uses the deep cascade structure to cascade different stages of HR and LR features to reconstruct HR images. However, it is neglected that when the HR image is reconstructed, the contribution of the HR features generated at different stages may be different, and the reconstructed HR is too smooth due to the increase of the network depth, and some high-frequency information is lost.

In order to reconstruct a clearer SR image of CMR images, we propose the multichannel residual attention network (MCRN); our contributions are three-fold:

1. We propose the multichannel residual dilated convolution structure by combining the idea of dilated convolution and residual learning, which can efficiently extract the multichannel contextual information of CMR image
2. We design the residual framework of long and short skip connections to improve the accuracy of image feature information acquisition
3. We introduce the attention mechanism to automatically allocate attention resources to the feature maps generated at each stage of the residual back-projection block and each channel of the feature map

## 2. Related Work

### 2.1. Residual Learning

When training a very deep network structure, since the initialization parameters are very close to zero, it is easy to cause gradient dispersion when the network reversely broadcasts the update parameters. This makes deepening the network structure not only unable to improve network performance but also even worse. In response to this problem, He et al. [19] proposed the residual net (ResNet), using the idea of residual learning to alleviate the problem of gradient dispersion. The main idea is to add a direct connection channel to the network, allowing a certain percentage of the previous network output to be retained. However, there are certain difficulties in learning identity mapping. To avoid learning the parameters of identity mapping, the ResNet uses the network structure shown in Figure 1, namely, *H*(*x*) = *F*(*x*) + *x*. It can be converted to *F*(*x*) = *H*(*x*) − *x*, where *F*(*x*) is the residual term. When the residual term is *F*(*x*) = 0, the identity mapping *H*(*x*) = *x* can be easily constructed. Compared to learning the identity mapping *H*(*x*) = *x*, learning *F*(*x*) = 0 is easier.

### 2.2. Deep Back-Projection Network

Haris et al. [18] proposed the deep back-projection networks (DBPN), which use an iterative back-projection method to learn the mapping relationship between LR and HR images and use an error feedback mechanism to correct the reconstruction between LR and HR images error. According to Figure 2, the DBPN algorithm contains several serial upsampling layers, and the spatial detail information in the picture is extracted through continuous degradation and SR reconstruction of the picture. For the input LR image, first perform initial feature extraction to obtain shallow features, and then use several iterative up-block and down-block to learn the reconstruction error between HR and LR features, and finally the HR feature maps generated in the previous stages are cascaded and the predicted image is reconstructed. In addition, each back-projection includes up-block and down-block operations, where up-block and down-block are implemented using a deconvolution layer and a convolution layer, respectively.

## 3. Methodology

Aiming at the problem of loss of feature information and gradient dispersion in the learning process caused by the deeper network structure, as can be seen from Figure 3, we propose the multichannel residual attention network structure, which mainly includes initial layer, multichannel up-block and down-block residual attention module (MCUD), residual attention module (RA), and reconstruction layer.

### 3.1. Multichannel Up-Block and Down-Block Residual Attention Modules

To solve the problem of high-frequency information loss the longitudinal deepening network, a multichannel residual cavity convolutional network was proposed, as shown in Figure 4. Combining the idea of dilated convolution and residual error, it can obtain the multichannel background information of CMR images more effectively. Furthermore, to increase the receptive field without pooling loss information, so that each convolution output contains a larger range of information, we have introduced dilated convolution in the multichannel up-block and down-block residual modules, the difference is that the dilated convolution uses expansion rates of 1, 3, and 5 to add different receptive fields, and the parameters are shown in Table 1.

Regarding the up-block module, the input of the up-block is the output of the down-block in the previous projection unit cascaded with this projection unit, that is, the input of *n* up-blocks is [*L*^1^, ⋯, *L*^*n*−1^], and then the input of the projection block is cascaded together using the cascade layer. At the same time, to reduce the amount of calculation, a convolutional layer with a convolution kernel size of 1∗1 is used to reduce the dimensionality of the feature map to obtain feature *L*^*n*−1^, and then perform upsampling and downsampling operations on *L*^*n*−1^ to obtain *H*_0_^*n*^ and *L*_0_^*n*^, respectively, and calculate *L*^*n*−1^ and *L*_0_^*n*^, and use *e*_*n*_^1^ to correct the mapping relationship between HR features and LR features.

The up-block module is defined as follows:

(1) $$\begin{array}{c} \text{Scale up}:H_{0}^{n}=\left(L^{n-1}*p_{n}\right){↑}^{s}, \end{array}$$

(2) $$\begin{array}{c} \text{Scale down}:L_{0}^{\text{n}}=\left(H_{0}^{n}*g_{n}\right){↓}_{s}, \end{array}$$

(3) $$\begin{array}{c} \text{Residual}:e_{n}^{l}=L_{0}^{n}-L^{n-1}, \end{array}$$

(4) $$\begin{array}{c} \text{Scake residual up}:H_{1}^{n}=\left(e_{n}^{1}*q_{n}\right){↑}^{s}, \end{array}$$

(5) $$\begin{array}{c} \text{Output feature map}:H^{n}=H_{0}^{n}+H_{1}^{n}. \end{array}$$

Regarding the down-block module, the input of the down-block is also the result of cascading the residual learning of the previous projection blocks of this projection unit, and the input feature information is sequentially cascaded and linearly mapped to obtain the feature map *H*^*n*^. Subsequently, the down- and upsampling operations are sequentially performed, and the reconstruction error *e*_*h*_^*n*^ is calculated, and the secondary reconstruction error is used to guide the reconstruction of the LR feature map.

The down-block module is defined as follows:

(6) $$\begin{array}{c} \text{Scale down}:L_{1}^{n}=\left(H_{2}^{n}*g_{n}\right){↓}_{s}, \end{array}$$

(7) $$\begin{array}{c} \text{Scale up}:H_{3}^{n}=\left(L_{1}^{n}*p_{n}\right){↑}^{s}, \end{array}$$

(8) $$\begin{array}{c} \text{Residual}:e_{h}^{n}=H_{3}^{n}-\left(H_{2}^{n}*k_{n}\right), \end{array}$$

(9) $$\begin{array}{c} \text{Scale residual up}:L_{2}^{\text{n}}=\left(e_{h}^{n}*g_{n}\right){↓}_{s}, \end{array}$$

(10) $$\begin{array}{c} \text{Output feature map}:L^{n}=L_{0}^{n}+L_{1}^{n}, \end{array}$$

where ∗ is the convolution operator, ↑^s^ and ↓_s_ are the upsampling and downsampling operations with scale factor *s*, respectively, *p*_*n*_ is the upsampling deconvolutional layer of the *n*-th up-block and down-block (UD), *g*_*n*_ is the downsampling convolutional layer of the *n*-th UD, *q*_*n*_ is 128-dimensional feature fusion layer of the *n*-th UD, and *k*_*n*_ denotes the *n*-th UD of 64-dimensional feature fusion layer [20] as shown in Figure 5.

### 3.2. Residual Attention Module

To better extract the feature information of the CMR image, the MCRN model deepens the number of network layers. Further, the residual attention module (RA) contains 3 residual attention block modules (RAB), and the network structure is shown in Figure 6. As the number of network layers deepens, the residual structure is introduced. There are two reasons for introducing the residual structure here: one is that the network deepening has network degradation problems, and learning residuals can reduce the impact of such problems in deep network training. Furthermore, since there are a lot of similar low-frequency information between HR images, using the residual structure can reduce repeated learning of similar low-frequency information, speed up the network convergence speed, and save computing time. Secondly, the attention mechanism is introduced to allocate different attention resources to the feature maps in different stages of interconnection and different channels of different feature maps, to learn deeper feature information.

### 3.3. Reconstruction Layer

In the high-power reconstruction part, first use 3∗3 convolution to sort and filter redundant information to reconstruct the optimal sparse network structure, and then use subpixel convolution to upsample *T* to the target multiple *γ*. Finally, the mapping from *I*^LR^ to *I*^SR^ is completed through a layer of 3∗3 convolution to generate a clear SR image; the specific formula is as follows:

(11) $$\begin{array}{c} I^{\text{SR}}=\sigma \;\omega_{3\times 3}^{l}\times \text{SF }\sigma \;\omega_{3\times 3}^{l-2}\times T+b^{l-2}+b^{l}, \end{array}$$

where *I*^SR^ represents the predicted HR image, the symbol × represents the convolution operator, the symbol + represents the pixel-by-pixel addition operator, SF *x* represents the subpixel convolution operation of rearranging the combined pixels, and the *l* in the variable superscript is the last one in the network convolutional layer and *l* − 2 is the first convolutional layer of the reconstruction part.

## 4. Experiment and Analysis

### 4.1. Dataset and Training Details

Owing to the relatively deep network, the algorithm needs to use a larger training set to train better results. T91 [21] dataset and Berkeley Segmentation Dataset 500 (BSD500) are selected, respectively, with a total of 591 images [5]. In order to make full use of the depth image, the dataset image is rotated by 90°, 180°, and 270° and scaled according to the coefficients of 0.9, 0.8, and 0.7 and then saved the picture; a total of 9456 images are generated; and the test dataset uses Set5 [20], Set14 [22], and Urban100 [23] datasets.

To build a CMR diagnosis model based on deep learning, we tested it on the public CMR datasets. We used the cardiac MRI dataset [24], which is the medical imaging data of atrium in patients with heart disease, including cardiac MR images of 33 subjects, with a total of 7980 images (Cardiac MRI dataset: http://www.cse.yorku.ca/~mridataset/).

Furthermore, our algorithm was trained on Ubuntu 16.04, CUDA Toolkit 10.0, PyTorch 1.20, python 3.7, and GPU NVIDIA GeForce RTX 1080Ti. In addition, the initial learning rate is set to 10^−4^, the Adam optimizer was set with*β*_1_ = 0.9,*β*_2_ = 0.999, *ε* = 10^−8^, and*L*_1_-normalization was used as the loss function. To evaluate the performance of the proposed MCRN, we use the peak signal-to-noise ratio (PSNR) [25] and structural similarity index (SSIM) [26] as the evaluating metrics. The specific operations of PSNR and SSIM are shown in Equations (12) and (13).

(12) $$\begin{array}{c} \text{PSNR}=10\text{l g}\frac{MN}{{\left\|I_{H}-I_{S}\right\|}^{2}}, \end{array}$$

where *M* and *N* represent the sizes of the HR image and the SR image.

(13) $$\begin{array}{c} \text{SSIM}=\frac{\left(2\mu_{H}\mu_{S}+C_{1}\right)\left(\sigma_{HS}+C_{2}\right)}{\left({\mu_{H}}^{2}+{\mu_{S}}^{2}+C_{1}\right)\left({\sigma_{H}}^{2}+{\sigma_{S}}^{2}+C_{2}\right)}, \end{array}$$

where *μ*_*H*_ and *μ*_*S*_ represent the average grey values of the HR image and the SR image, *σ*_*H*_ and *σ*_*S*_ represent the variances of the HR image and the SR image, and *σ*_*HS*_ denotes the covariance of the HR image and the SR image.

### 4.2. Comparison with Other State-Of-The-Art Algorithms

We compare our method with 9 state-of-the-art SR algorithms: Bicubic [6], A+ [27], SCN [28], SRCNN [9], FSRCNN [10], VDSR [11], DRCN [12], LapSRN [14], and DRRN [29].  Table 2 shows the comparison of experimental results with an amplification factor of 2, 3, and 4. It can be found from Table 2 that when the scaling factors are 2, 3, and 4, the algorithm proposed in this paper achieves the best performance in PSNR and SSIM on each dataset. When the scaling factor is 2, the algorithm in this paper achieves the optimal reconstruction effect for each index on each dataset. Among them, when the scaling factor is 2 on the Set14 dataset, the PSNR improvement of this algorithm is the most obvious compared with other algorithms. It reaches 33.72 dB, which is 0.40 dB higher than the PSNR of the suboptimal DRRN algorithm.

As can be seen from the Figure 7, the image reconstructed by Bicubic [3] appears severely blurred, and the details of CMR cannot be observed. The image reconstructed by SRCNN [9], FSRCNN [10], and LapSRN [15] appears severely distorted, and the details of the information are not enough. Moreover, the result of the reconstruction of VDSR [18], DRCN [13], and DRRN [19] algorithms obtains a better visual experience, and there is still a lack of detailed information. In fact, compared with state-of-the-art methods, our MCRN algorithm restores the details of the original image and improves the clarity of the CMR image, indicating that our model shows obvious superiority in both objective indicators and visual effects.

## 5. Conclusion

In this paper, we propose a CMR image superresolution algorithm based on multichannel residual attention network (MCRN), which mainly uses the back-projection method and combines residual learning and attention mechanisms to alleviate the problems of insufficient feature information and loss of high-frequency information in the learning process. At the same time, the difference between feature maps is fully utilized, so that more useful high-frequency information can be discovered when reconstructing the predicted image. The experimental results prove the superiority of the algorithm in the PSNR and SSIM indicators, and the detailed information of the predicted CMR image is more abundant, which effectively improves the clarity of the CMR image and can effectively assist the CMR diagnosis and quantitative evaluation. For future implementation, we will consider improving the image reconstruction part so that the reconstruction part can make full use of the characteristics of network learning and achieve the excellent image reconstruction effects.

## Figures and Tables

**Figure 1:** Structure of residual learning.

**Figure 2:** The architect of deep back-projection network.

**Figure 3:** The architect of multichannel residual attention network.

**Figure 4:** The architect of multichannel up-block and down-block residual modules.

**Figure 5:** Structure of up- and down-block modules.

**Figure 6:** Structure of residual attention module.

**Figure 7:** Comparison of rendering of images with superresolution magnification of 4 under our MCRN and other state-of-art methods. (a) Aorta in short axis orientation (3 × 11 × 25, coronal), (b) aorta in short axis orientation (3 × 11 × 25, axial), and (c) heart imaged in 3 orthogonal orientations (axial).

**Table 1:** The feature size of the MCRN for CMR images SR.

Network components	Kernel size	Stride	Padding	Input size	Output size
Initial layer	3∗3	1	1	H∗W∗1	H∗W∗64

RAB					
Conv 1	3∗3	1	1	H∗W∗64	H∗W∗64
Conv 2	1∗1	1	0	H∗W∗64	H∗W∗4
Conv 3	1∗1	1	0	H∗W∗4	H∗W∗64

Up-block					
DeConv	4∗4	2	1	H∗W∗64	H∗W∗128
Conv	4∗4	2	1	H∗W∗128	H∗W∗64
DeConv	4∗4	2	1	H∗W∗64	H∗W∗128

Down-block					
Conv	4∗4	2	1	H∗W∗128	H∗W∗64
DeConv	4∗4	2	1	H∗W∗64	H∗W∗128
Conv	4∗4	2	1	H∗W∗128	H∗W∗64

Middle layer	3∗3	1	1	H∗W∗64	H∗W∗64

Upsample	3∗3	1	1	H∗W∗64	2H∗2 W∗64

Reconstruction layer	3∗3	1	1	2H∗2 W∗64	2H∗2 W∗1

**Table 2:** Average PSNR/SSIM of various SSIR methods; the best and second-best results are in bold and italics.

Algorithm	Scale	Set 5		Set 14		Urban 100	
		PSNR	SSIM	PSNR	SSIM	PSNR	SSIM
Bicubic [6]	2×	33.69	0.931	30.25	0.870	26.88	0.841
A+ [27]	2×	36.60	0.955	32.32	0.906	29.25	0.895
SCN [28]	2×	36.58	0.954	32.35	0.905	29.52	0.897
SRCNN [9]	2×	36.72	0.955	32.51	0.908	29.53	0.896
FSRCNN [10]	2×	37.05	0.956	32.66	0.909	29.88	0.902
VDSR [11]	2×	37.53	*0.959*	33.05	0.913	30.77	*0.914*
DRCN [12]	2×	37.63	*0.959*	33.06	0.912	30.76	*0.914*
LapSRN [14]	2×	37.52	*0.959*	33.08	0.913	30.41	0.910
DRRN [29]	2×	*37.74*	*0.959*	*33.23*	*0.914*	*31.23*	**0.919**
MCRN (ours)	2×	**37.88**	**0.961**	**33.63**	**0.919**	**31.27**	**0.919**

Bicubic [6]	3×	30.41	0.869	27.79	0.775	24.46	0.735
A+ [27]	3×	32.62	0.909	29.15	0.820	26.05	0.799
SCN [28]	3×	32.62	0.908	29.16	0.818	26.21	0.801
SRCNN [9]	3×	32.78	0.909	29.32	0.823	26.25	0.801
FSRCNN [10]	3×	33.18	0.914	29.37	0.824	26.43	0.808
VDSR [11]	3×	33.67	0.921	29.78	0.832	27.14	0.829
DRCN [12]	3×	33.83	0.922	29.77	0.832	27.15	*0.828*
LapSRN [14]	3×	33.82	0.922	29.87	0.832	27.07	*0.828*
DRRN [29]	3×	**34.03**	*0.924*	*29.96*	*0.835*	**27.53**	0.764
MCRN (ours)	3×	*33.99*	**0.925**	**30.28**	**0.844**	*27.27*	**0.830**

Bicubic [6]	4×	28.43	0.811	26.22	0.715	23.14	0.658
A+ [27]	4×	30.32	0.860	27.34	0.751	24.34	0.721
SCN [28]	4×	30.41	0.863	27.39	0.751	24.52	0.726
SRCNN [9]	4×	30.50	0.863	27.52	0.753	24.53	0.725
FSRCNN [10]	4×	30.72	0.866	27.61	0.755	24.62	0.728
VDSR [11]	4×	31.35	0.883	28.02	0.768	25.18	0.754
DRCN [12]	4×	31.54	0.884	28.03	0.768	25.14	0.752
LapSRN [14]	4×	31.54	0.885	28.19	*0.772*	25.21	0.756
DRRN [29]	4×	**31.68**	**0.888**	*28.21*	*0.772*	**25.44**	**0.764**
MCRN(ours)	4×	*31.67*	*0.887*	**28.45**	**0.783**	*25.25*	*0.759*

## Data Availability

The image data used to support the findings of this study have been deposited in the Cardiac MRI Dataset repository (http://www.cse.yorku.ca/~mridataset/) and AMRG Cardiac Atlas repository (http://www.cardiacatlas.org/studies/amrg-cardiac-atlas/).
